The article "Curcumin Potentiates Rhabdomyosarcoma Radiosensitivity by Suppressing NF-κB Activity" was retracted in 2019. Reasons: fabricated or falsified data; manipulated images; duplicated images.

# Curcumin Potentiates Rhabdomyosarcoma Radiosensitivity by Suppressing NF-κB Activity

**DOI:** 10.1371/journal.pone.0051309

**Published:** 2013-02-07

**Authors:** W. Shannon Orr, Jason W. Denbo, Karim R. Saab, Catherine Y. Ng, Jianrong Wu, Kui Li, Jo Meagan Garner, Christopher L. Morton, Ziyun Du, Lawrence M. Pfeffer, Andrew M. Davidoff

**Affiliations:** 1 University of Tennessee Health Science Center, Department of Surgery, Memphis, Tennessee, United States of America; 2 St. Jude Children's Research Hospital, Department of Surgery, Memphis, Tennessee, United States of America; 3 St. Jude Children's Research Hospital, Department of Biostatistics, Memphis, Tennessee, United States of America; 4 University of Tennessee Health Science Center, Department of Microbiology, Immunology and Biochemistry, Memphis, Tennessee, United States of America; 5 University of Tennessee Health Science Center, Department of Pathology and the Center for Cancer Research, Memphis, Tennessee, United States of America; Johns Hopkins University, United States of America

## Abstract

Ionizing radiation (IR) is an essential component of therapy for alveolar rhabdomyosarcoma. Nuclear factor-kappaB (NF-κΒ) transcription factors are upregulated by IR and have been implicated in radioresistance. We evaluated the ability of curcumin, a putative NF-κΒ inhibitor, and cells expressing genetic NF- κΒ inhibitors (IκBα and p100 super-repressor constructs) to function as a radiosensitizer. Ionizing radiation induced NF-κΒ activity in the ARMS cells *in vitro* in a dose- and time-dependent manner, and upregulated expression of NF-κΒ target proteins. Pretreatment of the cells with curcumin inhibited radiation-induced NF-κΒ activity and target protein expression. *In vivo*, the combination of curcumin and IR had synergistic antitumor activity against Rh30 and Rh41 ARMS xenografts. The greatest effect occurred when tumor-bearing mice were treated with curcumin prior to IR. Immunohistochemistry revealed that combination therapy significantly decreased tumor cell proliferation and endothelial cell count, and increased tumor cell apoptosis. Stable expression of the super-repressor, SR-IκBα, that blocks the classical NF-κB pathway, increased sensitivity to IR, while expression of SR-p100, that blocks the alternative pathway, did not. Our results demonstrate that curcumin can potentiate the antitumor activity of IR in ARMS xenografts by suppressing a classical NF-κΒ activation pathway induced by ionizing radiation. These data support testing of curcumin as a radiosensitizer for the clinical treatment of alveolar rhabdomyosarcoma.

**Impact of work:**

The NF-κΒ protein complex has been linked to radioresistance in several cancers. In this study, we have demonstrated that inhibiting radiation-induced NF-κΒ activity by either pharmacologic (curcumin) or genetic (SR-IκBα) means significantly enhanced the efficacy of radiation therapy in the treatment of alveolar rhabdomyosarcoma cells and xenografts. These data suggest that preventing the radiation-induced activation of the NF-κΒ pathway is a promising way to improve the antitumor efficacy of ionizing radiation and warrants clinical trials.

The article "Curcumin Potentiates Rhabdomyosarcoma Radiosensitivity by Suppressing NF-κB Activity" was retracted in 2019. Reasons: fabricated or falsified data; manipulated images; duplicated images.

## Introduction

Rhabdomyosarcoma (RMS) is the most common soft tissue sarcoma of childhood [1]. There are two main histologic subtypes of RMS, embryonal (ERMS) and alveolar (ARMS). ARMS accounts for only 20–30% of newly diagnosed RMS in children but is associated with a much poorer prognosis [2]. An analysis of patients with nonmetastatic RMS from the Intergroup Rhabdomyosarcoma Studies (IRS) indicates a 5-year failure-free survival of only 65% for ARMS, despite intensive therapy; the outcome for patients presenting with metastatic ARMS is much worse [2]. Multimodal treatment of ARMS consists of surgical resection, systemic chemotherapy and ionizing radiation (IR). Findings from the IRS support the use of IR for all ARMS, regardless of stage and grade [3].

Although ionizing radiation is a critical component of RMS therapy, it is associated with significant early and late complications. Early complications such as inflammation can occur within hours to several weeks after therapy. Changes in cell membrane permeability and histamine release subsequently lead to cell loss, causing mucositis and epidermal desquamation. Late effects of ionizing radiation include cognitive defects, hypothyroidism, musculoskeletal deformities, pulmonary fibrosis, cardiac dysfunction and second malignancies [4]–[8]. Since the adverse effects of radiation are dose-dependent, increasing the efficacy of ionizing radiation on a per dose basis could limit its toxic side effects.

The nuclear factor-kappaB (NF-κΒ) family of transcription factors regulate the expression of genes involved in immune and inflammatory responses, developmental processes, and cellular proliferation and apoptosis [9]. Inhibitory IκB proteins tightly regulate NF-κΒ activity [10]. The classical NF-κΒ pathway involves serine phosphorylation and degradation of IκB proteins leading to the dissociation of the cytosolic inactive NF-κΒ/IκB complexes, and subsequent NF-κΒ translocation into the nucleus for DNA binding. However, a growing number of NF-κB inducers activate an alternative NF-κB pathway that does not involve IκB degradation, but rather involves the ubiquitination and proteolytic processing of p100/NFKB2 protein and nuclear translocation of p52:RelB dimers to regulate specific NF-κB target genes [9], [11]. Induction of NF-κB has been linked to tumor cell proliferation, angiogenesis, and inhibition of apoptosis, metastasis and radioresistance [12], [13].

The article "Curcumin Potentiates Rhabdomyosarcoma Radiosensitivity by Suppressing NF-κB Activity" was retracted in 2019. Reasons: fabricated or falsified data; manipulated images; duplicated images.

Curcumin (diferuloylmethane), a yellow-colored polyphenol, is an active component of *Curcuma longa*, commonly known as turmeric. Curcumin has been shown to suppress NF-κΒ activation and down-regulate expression of NF-κΒ gene targets [13]–[17]. Curcumin has also been shown to sensitize colorectal cancer cells and neuroblastoma cells to ionizing radiation *in vitro* by inhibiting induction of NF-κΒ activity [18], [19]. Curcumin has been shown to be to be nontoxic in clinical trials with doses as high as 12 gm/day [20].

Despite advances in multi-modality therapy, many children with ARMS face a poor prognosis and so new treatment strategies are desperately needed. In this study, we tested the ability of curcumin to inhibit NF-κΒ activity and to act as a radiosensitizer. Our studies demonstrate that curcumin can potentiate the antitumor effects of ionizing radiation *in vitro* and in orthotopic alveolar rhabdomyosarcoma xenografts in mice.

## Methods

### Cell lines

The human alveolar rhabdomyosarcoma-derived cell lines, Rh30 and Rh41, were established at St. Jude Children's Research Hospital, Memphis, TN by Dr. Peter Houghton (Columbus, OH). The handling of these two cell lines in this manner has been supported by the St. Jude Children's Research Hospital IRB. Cells that stably express the IκBα and p100 super-repressors were made by selecting blastocidin-resistant cell populations following transduction with retroviral vectors encoding either an Iκβα mutant (SR-IκBα), a p100 mutant (SR-p100), or empty vector (EV). The constructs encoding the IκBα and p100 mutants were kindly provided by Dr. Jiandong Li (Atlanta, GA) and Dr. Shao-Cong Sun (Houston, TX), respectively.

### Curcumin preparation

A liposomal formulation of curcumin was prepared to improve the delivery of the drug. 1, 2-Dimyristoyl-sn-glycero-3-phosphocholine (DMPC) and 1, 2-dimyristoylsn-glycero-3-[phosphor-rac- (1-glycerol)] (DMPG) were obtained from Avanti Polar Lipids (Alabaster, AL). Curcumin (ACROS, Morris Plains, NJ), dimethylsulfoxide (DMSO), and tert-butanol were obtained from Sigma Chemical Company (St. Louis, MO). Lyophilization of curcumin involved several steps. A 10∶1 total lipid to curcumin ratio (weight/weight) was used [21]. Curcumin was dissolved in DMSO at 50 mg/ml and the lipid (9∶1, DMPC:DMPG) was dissolved at 20 mg/ml in tert-butanol. Aliquots of this solution were then lyophilized to remove all DMSO and tert-butanol. The lyophilized powder was stored at −20°C and then reconstituted in normal saline for use.

The article "Curcumin Potentiates Rhabdomyosarcoma Radiosensitivity by Suppressing NF-κB Activity" was retracted in 2019. Reasons: fabricated or falsified data; manipulated images; duplicated images.

### Cell viability analysis

The effects of curcumin and IR on cell viability were determined by an Alamar Blue viability assay (Invitrogen, Carlsbad, CA), according to the manufacturer's instructions. Cells were irradiated with a cesium-137 source and/or treated with liposomal curcumin. Alamar blue was added to treated cells and after 4 hours the absorbance was read on a Synergy 2 Multi-Mode Microplate Reader (Biotek, Winooski, VT). These experiments were performed in triplicate.

### Apoptosis

To analyze the effects of curcumin on apoptosis, cells were treated with 10 μmol of liposomal curcumin for 24 hours before irradiation. Cells were analyzed by flow cytometry for apoptosis (Annexin V staining) at 48 hours following irradiation.

### NF-κB DNA binding assays

Nuclear extracts were prepared using the Affymetrix Nuclear Extraction Kit (Affymetrix, Santa Clara, CA) and stored at −80°C. To determine NF-κΒ DNA binding activity, an electrophoretic mobility shift assay (EMSA) was performed on nuclear extracts following the protocol by Promega Gel Shift Assay Systems. In brief, nuclear extracts were incubated with a ^32^P-end-labeled double-stranded NF-κΒ oligonucleotide containing a tandem repeat consensus sequence of 5′-AGT TGA GGG GAC TTT CCC AGG C-3′, and separated by electrophoresis on 4% polyacrylamide gels. Bands were visualized on PhosphorImager and quantified with ImageQuant 5.2 software (Molecular Dynamics, Sunnyvale, CA).

### Western blot analysis

Antibodies for matrix metalloproteinase-9 (MMP-9), IκBα, and pIκBα were obtained from Santa Cruz Biotechnology, Santa Cruz, CA. Antibodies for bcl-2 and XIAP were obtained from Cell Signaling (Danvers, MA). Antibodies for Cox-2 were obtained from Cayman Chemical (Ann Arbor, MI). Protein expression of MMP-9, Cox-2, bcl-2, XIAP, IκBα and pIκBα was determined by western blot analysis as previously described [22].

### Murine ARMS tumor model

All murine experiments were done in accordance with a protocol approved by the Institutional Animal Care and Use Committee of St. Jude Children's Research Hospital. Orthotopic intramuscular (IM) ARMS xenografts were established in male CB-17 severe combined immunodeficient mice (Taconic, Hudson, NY), as previously described [23]. The size of the IM tumors was estimated by measuring the volume of the normal left calf and subtracting that from the volume of the tumor-bearing right calf. Measurements were done weekly using handheld calipers, and volumes calculated as width^2^ x length x 0.5. Mice with size-matched Rh30 or Rh41 xenografts were placed into one of four groups approximately 4 weeks after tumor cell injection and then treated with empty liposome given intraperitoneally (IP), 50 mg/kg liposomal curcumin IP daily until sacrifice, 10 Gy IR, or combination therapy. A single dose of 10 Gy IR was administered using an Orthovoltage D3000 x-ray tube (Gulmay Medical Ltd, Surrey, UK) [23]. A lead shield with a 2 cm hole was used to deliver radiation to the tumor while protecting the mice from radiation. Four mice in each group were sacrificed for tumor analysis 4 hr after radiation. The remaining mice were sacrificed approximately 3 weeks following the start of treatment.

The article "Curcumin Potentiates Rhabdomyosarcoma Radiosensitivity by Suppressing NF-κB Activity" was retracted in 2019. Reasons: fabricated or falsified data; manipulated images; duplicated images.

In addition, we examined the response *in vivo* of Rh30 cell lines that express the SR-IκBα or SR-p100 super-repressor construct. Xenografts of Rh30-EV, Rh30 SR-IκBα, and Rh30 SR-p100 were established in the right calf of mice. For each xenograft, mice were placed into 2 groups of equivalent tumor burden to receive 10 Gy IR or to serve as controls.

### Immunohistochemistry

Formalin-fixed, paraffin-embedded, 4-μm thick tumor sections were stained with rat anti-mouse CD34 (RAM 34; PharMingen, San Diego, CA) antibodies as previously described [24]. Apoptosis in tumors was determined by terminal deoxynucleotidyl transferase-mediated dUTP nick end labeling using a commercially available *in situ* apoptosis detection kit (Serologicals, Billerica, MA) as previously described [23]. Tumor cell proliferation was analyzed by staining with an anti-Ki67 antibody (rabbit monoclonal clone SP6; Neomarkers, Fremont, CA). Results were expressed as the percentage of Ki-67 positive cells ± SE per 400x magnification as previously described [23].

### Statistical analysis

Isobolograms were used to assess the in vitro synergy between curcumin and radiation [25], [26]. A weighed nonlinear dose-response model [26] using SAS NLIN procedure was used to fit fluorescence emission intensity data. Observed three-dimensional dose-response plots, fitted dose-response plotsand isobolograms were generated. Dose-independent synergy of combined curcumin and radiation was estimated from the model by the non-additivity parameter, α, which indicates synergism (α>0), antagonism (α<0), or no interaction (α = 0). For *in vivo* experiments, Bliss's independent joint action principle was used to define a synergy index (SI). Continuous variables are reported as mean ± SEM and were compared using an unpaired Student's *t* test with a p-value <.05 considered significant. Data were analyzed and graphed using Sigma Plot (Version 9; SPSS Inc, Chicago, IL).

## Results

### Ionizing radiation induces NF-κB activation in alveolar rhabdomyosarcoma cells in a dose- and time-dependent manner through the canonical pathway

To determine NF-κΒ DNA binding activity in Rh30 and Rh41 cells exposed to ionizing radiation (10 Gy), nuclear extracts were prepared at various times after irradiation and analyzed by electrophoretic mobility shift assay (EMSA). Both cell lines showed a time-dependent induction of NF-κΒ DNA binding activity, with activity evident within 1 hr after radiation exposure, and reaching a maximum activity at ∼2 hr (Fig. 1A). To further characterize the induction of NF-κΒ DNA binding activity, Rh30 and Rh41 cell lines were exposed to varying radiation doses (0–10 Gy) for 2 hr and nuclear extracts were prepared. In both cell lines, ionizing radiation activated NF-κΒ in a dose-dependent manner, with marked induction occurring at 10 Gy (Fig. 1B). Supershift assays were then performed with antibodies directed to specific NF-κΒ subunits to determine which NF-κΒ proteins comprised the radiation-induced complex. These assays showed that the p50 and p65 subunits comprise the radiation-induced NF-κΒ complex (Fig. 1C).

The article "Curcumin Potentiates Rhabdomyosarcoma Radiosensitivity by Suppressing NF-κB Activity" was retracted in 2019. Reasons: fabricated or falsified data; manipulated images; duplicated images.

**Figure 1:** NF-κB induction by IR is dose- and time-dependent via the canonical pathway. (A) Ionizing radiation induces NF-κB in a time dependent manner. Rhabdomyosarcoma cell lines (Rh30 and Rh41) were exposed to 10 Gy radiation and nuclear extracts were harvested at various time points. In both cell lines, NF-κB activation, judged by EMSA showed maximal activity at 2 hrs (B) Ionizing radiation induction of NF-κB is dose dependent. In both cell lines, the maximum induction of NF-κB was seen at 10 Gy. (C) Ionizing radiation induces NF-κB activation via the classical pathway. Antibody super-shifts were performed with antibodies directed to specific NF-κB subunits. In both cell lines, the p50 and p65 subunits were the principal components of NF-κB activation. (D) IκBα super-repressor blocks NF-κB induction. Rh30 and Rh41 cell lines were transduced to express IκBα and p100 super-repressors. Radiation induced NF-κB activity in the empty vector and SR-p100 cell lines, but not in the SR- IκBα cell line. (E) IκBα and p100 super-repressor cell lines. TNFα (10 ng/ml for 1 hr) and LIGHT, also known as TNSF14, (10 ng/ml for 24 hr) were used to assess the activity of the super-repressor constructs on the classical and alternative NF-κB pathways, respectively. Expression of the SR- IκBα blocked TNFα stimulated NF-κB activity, expression of SR-p100 blocked LIGHT stimulated NF-κB activity.

The p50:p65 complex of NF-κΒ is induced through activation of the classical NF-κΒ pathway, which involves IκBα serine phosphorylation, polyubiqitination and subsequent proteosomal degradation. Therefore, expression of a mutant IκBα construct, in which the inducible serine phosphorylation sites have been mutated to alanine, should block classical NF-κΒ activation. In the alternative pathway, activation of the NF-κΒ-inducing kinase leads to proteolysis of p100 and liberation of the p52 complexes. A mutant p100 construct, in which the inducible serine phosphorylation sites have been mutated to alanine, should block the activation of the alternative NF-κΒ pathway. To determine whether radiation-induced NF-κΒ activation in ARMS cells involved the classical or alternative pathway, EMSA was performed on nuclear extracts prepared from ARMS cells that expressed IκBα and p100 super-repressors, respectively. As shown in Figure 1D, while radiation induced NF-κΒ activation in both Rh30 and Rh41 cell lines that express the empty vector or the SR-p100, expression of the SR-IκBα blocked the radiation-induced activation of NF-κΒ. The function of the IκBα and p100 constructs in the Rh30 cell line was confirmed by treatment with TNF-α (inducer of the classical NF-κΒ pathway) and by LIGHT (homologous to Lymphotoxin; inducer of alternative NF-κΒ activity) (Fig. 1E). [9], [11], [27] Taken together these results indicate that radiation-induced activation of NF-κΒ is both time- and dose-dependent, and involves the classical NF-κΒ pathway.

The article "Curcumin Potentiates Rhabdomyosarcoma Radiosensitivity by Suppressing NF-κB Activity" was retracted in 2019. Reasons: fabricated or falsified data; manipulated images; duplicated images.

### Curcumin suppresses radiation-induced NF-κB activation in alveolar rhabdomyosarcoma cells and sensitizes them to ionizing radiation by potentiating the apoptotic and cell cycle effects of IR

ARMS cells were treated with curcumin, a pharmacological inhibitor of NF-κΒ activity, to determine whether curcumin could abrogate the radiation-induced activation of NF-κΒ. Rh30 and Rh41 cells were pretreated with varying doses of liposomal curcumin (10, 25 and 50 µM) for varying lengths of time (0, 3 and 24 hr) prior to receiving a single dose of 10 Gy IR. Nuclear extracts were prepared 2 hr following radiation and assayed for NF-κΒ DNA binding activity by EMSA. As shown in Fig. 2, pretreatment for 24 hr with curcumin at all concentrations tested inhibited radiation-induced NF-κΒ activity in Rh30 and Rh41 cells. In addition, induction of NF-κΒ activity was also blocked when Rh41 cells were pretreated with 50 µM of curcumin for 3 hr prior to radiation.

**Figure 2:** Curcumin blocks radiation induced NF-κB induction in rhabdomyosarcomas. Rh30 and Rh41 cell lines were pretreated with varying doses of curcumin (10, 25 and 50 µM) for various lengths of time (0, 3 and 24 hrs) before exposure to radiation. EMSA was performed 2 hours following exposure to radiation to determine NF-κB activity. Pretreatment with curcumin for 24 hrs blocked the induction of NF-κB activity in both cell lines. In the Rh41 cell lines, NF-κB activity was blocked when 50 µM of curcumin was added 3 hrs before radiation treatment.

The article "Curcumin Potentiates Rhabdomyosarcoma Radiosensitivity by Suppressing NF-κB Activity" was retracted in 2019. Reasons: fabricated or falsified data; manipulated images; duplicated images.

We next sought to determine the effects of curcumin and IR on the proliferation of the ARMS cell lines. Liposomal curcumin inhibited the proliferation of Rh30 and Rh41 cells in a dose-dependent manner. The IC_50_ for inhibition of cell proliferation by curcumin was similar in both cell lines (17.5±1.92 µM for Rh30 to 19.3±1.89 µM for Rh41) (Fig. S1A). The anti-proliferative effects of liposomal curcumin were equivalent to that of free curcumin (IC_50_ 12.4±1.83 μmol and 15.32±1.67 µM for Rh30 and Rh41, respectively), confirming that there was no loss in the potency of curcumin during liposomal formulation. Treatment with empty liposomes alone had no effect on the proliferation of the rhabdomyosarcoma cell lines (data not shown). IR inhibited proliferation of Rh30 and Rh41 cells, in a dose dependent manner as well. The IC_50_ doses varied from 18.3±1.3Gy for Rh30 to 18.9±1.2Gy for Rh41 (Fig. S1B)

To test the effects of combination therapy, cells were pretreated with varying doses of curcumin for 24 hr prior to exposure to varying doses of radiation and cell viability was assessed at 96 hr following curcumin administration. The potential synergy between curcumin and radiation, on cell viability was assessed by an isobologram based-approach (Fig. S1C). (25, 26) A weighted non-linear dose-response model was fitted and the synergy of curcumin and radiation used in combination was estimated by the model non-additivity parameter (α). Curcumin and radiation showed synergy against the Rh30 and Rh41 cell lines. Treatment of Rh30 cells resulted in a positive non-additivity parameter of 5.54 with a 95% confidence interval (3.87, 7.20) that does not include 0. Treatment of Rh41 cells resulted in a non-additivity parameter of 5.86 with a 95% confidence interval (4.55, 7.17), which also does not include 0. Thus, we conclude that there was synergism between curcumin and radiation treatments in the Rh30 and Rh41 cell lines.

Cells were next treated with 10 µM liposomal curcumin (24 hr) prior to radiation exposure (10 Gy) and then analyzed by FACS for apoptosis by Annexin V-staining 48 hr after irradiation. The combination of curcumin and radiation significantly increased apoptosis compared to control in both cell lines. Apoptosis in control Rh30 cells was 4.6%±0.41 as compared to 8.67%±0.64 or 7.5%±0.3 in cells treated with radiation, or curcumin alone, respectively. In contrast apoptosis in Rh30 cells treated with a combination of radiation and curcumin was 19.5%±0.54 (p = .00003). A similar trend was observed in Rh41 cells. Apoptosis in control cells was 6.63%±0.66 as compared to 10.1%±1.6, or 9.9%±0.8 in cells treated with radiation or curcumin alone, while the combination of radiation and curcumin resulted in 22.9%±1.5 apoptosis (p = .0001) (Fig. S2A).

The article "Curcumin Potentiates Rhabdomyosarcoma Radiosensitivity by Suppressing NF-κB Activity" was retracted in 2019. Reasons: fabricated or falsified data; manipulated images; duplicated images.

### Curcumin inhibits degradation of IκBα in vitro

Since the classical NF-κΒ pathway involves the degradation of IκB, we investigated whether radiation induced IκBα degradation in IR-treated rhabdomyosarcoma cells. Whole cell extracts were prepared from Rh30 and R41 cells at various times after radiation exposure (10 Gy). Western blot showed IR induced a decrease in cellular IκBα levels within 1 hr and IκBα levels returned to control levels by 4 hr (Fig 3A). Treatment with curcumin suppressed the radiation-induced decrease in IκBα levels and phosphorylation of IκBα in Rh30 and Rh41 cells (Fig. 3B). These data demonstrate that curcumin inhibits radiation-induced NF-κΒ activation by suppressing the phosphorylation and degradation of IκBα in rhabdomyosarcomas.

**Figure 3:** Curcumin inhibits radiation induced degradation of IκBα in vitro. (A) Western blot showing radiation induces degradation of Iκβα in a time dependent manner in both Rh30 and Rh41 cell lines. (B) Curcumin pretreatment suppresses radiation-induced degradation of IκBα and phosphorylation of IκBα in Rh30 an Rh41.

### Curcumin inhibits radiation-induced NF-κB dependent genes involved in proliferation, metastasis, and anti-apoptosis

NF-κΒ has been shown to regulate the expression of target genes involved in proliferation (cyclin D1), inflammation (COX-2), metastasis (MMP-9), and anti-apoptosis (XIAP and Bcl-2). We next performed western blot analysis to determine whether curcumin modulated these target proteins in rhabdomyosarcoma cells treated with IR. This analysis revealed that, while radiation induced the expression of cyclin D1, COX-2, MMP-9, XIAP, and Bcl-2, curcumin treatment suppressed their induction by radiation (Fig. S3).

### SR-IκBα potentiates the antiproliferative and apoptotic effects of radiation

To further demonstrate the functional role of the radiation-induced canonical NF-κΒ pathway, the effect of IR on proliferation of Rh30 and Rh41cells expressing the IκBα super-repressor was analyzed. The Rh30 and Rh41 cells expressing the IκBα super-repressor were significantly more sensitive to the antiproliferative effects of 10 Gy IR when compared to the control (empty-vector expressing) cells and cells expressing the p100 super-repressor. The proliferation of irradiated Rh30 EV and Rh30 SR-p100 cell lines was 85.73±1.38% and 84.62±0.9% of control non-irradiated cells, respectively, as compared to 71.48±0.9% in the irradiated Rh30 cells expressing SR- IκBα (p = 0.0002). The proliferation of irradiated Rh41 EV and Rh41 SR-p100 cell lines was 81.66±0.53% and 80.63±0.44% of control nonirradiated cells, respectively, as compared to 68.93±1.7% in the Rh41 SR- IκBα cell line (p = 0.0002) (Fig. S4A).

The article "Curcumin Potentiates Rhabdomyosarcoma Radiosensitivity by Suppressing NF-κB Activity" was retracted in 2019. Reasons: fabricated or falsified data; manipulated images; duplicated images.

The effects of the NF-κΒ super-repressors were also analyzed by Annexin V-staining 48 hr after irradiation. Both Rh30 and Rh41 SR-IκBα cells had a significantly increased number of apoptotic cells compared to empty vector after exposure to 10 Gy radiation. The Rh30 EV and SR-p100 cell line had 10.87±0.9% and 11.73±1.5% Annexin V positive cells, respectively, as compared to 24.56±2.2% for the IκBα super-repressor cell line. The Rh41 EV and SR-p100 cell line had 11.66±0.9% and 12.8±0.5% Annexin V positive cells, respectively, as compared to 21.3±1.5% Annexin V positive cells in the IκBα super-repressor cell line (p = 0.0007) (Fig. S4B).

### Curcumin and radiation have synergistic antitumor activity against ARMS xenografts

We next determined whether curcumin sensitized rhabdomyosarcoma to IR *in vivo*. An orthotopic model of Rh30 and Rh41 ARMS was established in the right calf of CB-17 severe combined immunodeficient mice. After ∼1 month, mice with established xenografts were size-matched by tumor volume into 4 groups (n = 9/group). Mice received lyophilized vehicle IP daily, 50 mg/kg lyophilized curcumin IP daily, a single dose of 10 Gy IR, or combination therapy. A single dose of 10 Gy IR was given on day 7 of curcumin treatment for the group receiving combination therapy. Curcumin treatment was continued until mice were sacrificed. Following 3 weeks of treatment, the combination of curcumin and radiation had synergistic antitumor activity in the Rh30 xenografts (synergistic index  = −0.940, SE 0.072, 95% confidence interval −1.080, −0.799). The combination group had a tumor burden of 201.8±19.33 mm^3^ compared to 786±44.4 mm^3^, 679±51.46 mm^3^, and 1033.4±89.71 mm^3^ for the curcumin, radiation and control groups, respectively. Combination therapy in the Rh41 xenografts was also synergistic (synergistic index  = −0.915, SE 0.141, 95% confidence interval −1.192, −0.638). The combination group had a tumor burden of 275.1±55.9 mm^3^ compared to 927.4±98.7 mm^3^, 904.9±94.2 mm^3^and 1221.7±232.4 mm^3^ for the curcumin, radiation and control groups, respectively (Fig. 4A).

**Figure 4:** Curcumin and Radiation have synergistic antitumor activity against ARMS xenografts. (A) The combination of curcumin and radiation had synergistic antitumor activity in the Rh30 xenografts (synergistic index  = −0.940, SE 0.072, 95% confidence interval −1.080, −0.799). In the Rh41 cell line, the combination of curcumin and radiation was also synergistic (synergistic index  = −0.915, SE 0.141, 95% confidence interval (−1.192, −0.638). (B) The antitumor activity when curcumin was given either concomitantly with or prior to radiation.

The article "Curcumin Potentiates Rhabdomyosarcoma Radiosensitivity by Suppressing NF-κB Activity" was retracted in 2019. Reasons: fabricated or falsified data; manipulated images; duplicated images.

We next confirmed the importance of the timing of curcumin administration on the effectiveness of radiation exposure. Rh30 and Rh41 tumors were established and mice were size-matched into 3 groups (n = 5). Mice received lyophilized vehicle IP daily, 10 Gy radiation followed immediately by 50 mg/kg liposomal curcumin IP daily, and 10 Gy radiation 7 days after the start of liposomal curcumin. Curcumin was continued until the animals were sacrificed. In both rhabdomyosarcoma xenografts, the effect of the timing of curcumin treatment prior to irradiation was found to be critical. In the Rh30 cell line, the group that received radiation before curcumin administration had a tumor volume of 620±68.5 mm^3^ compared to 242±27.5 mm^3^ for the group that was pretreated with curcumin before radiation (p = 0.0017). In the Rh41 cell line, the group that received radiation before curcumin administration had a tumor volume of 756±92.4 mm^3^ compared to 227±26.4 mm^3^ for the group that was pretreated with curcumin before radiation (p = 0.0003) (Fig. 4B). These results confirm that timing of curcumin administration is critical when attempting to maximize the anti-tumor effect of combination therapy.

### Curcumin suppresses radiation-induced NF-κB activation in vivo

We performed EMSA to determine NF-κΒ activity in tumors harvested 4 hours after radiation therapy. EMSA confirmed that radiation induced NF-κΒ activation in both Rh30 and Rh41 xenografts and that pre-treatment with curcumin inhibited this radiation-induced NF-κΒ activation (Fig. 5A). As was done previously in our *in vitro* studies, we performed western blot analysis for IκBα from tumor tissues harvested post-IR to determine the mechanism whereby curcumin inhibits NF-κΒ activation *in vivo*. This analysis showed that in both rhabdomyosarcoma xenografts, radiation-induced NF-κΒ activation was mediated by IκBα degradation (Fig. 5B), and IκBα degradation was abrogated by curcumin.

**Figure 5:** Curcumin treatment suppresses radiation-induced NF-κB activation in vivo. Xenograft tumors were harvested 4 hr after radiation therapy. (A) EMSA revealed that in both the Rh30 and Rh41 curcumin suppressed radiation-induced activation of NF-κβ. (B) Western blot analysis revealed radiation-induced degradation and increased phosphorylation of IκBα which was suppressed by curcumin.

### Curcumin enhances the effect of radiation on tumor cell proliferation and apoptosis

To investigate the mechanism of synergy, we examined the effects of curcumin and radiation on tumor cell proliferation and apoptosis by Ki67 and TUNEL immunohistochemical staining, respectively. In both rhabdomyosarcoma xenografts, the percentage of proliferating cells was significantly decreased in the combination therapy. In the Rh30 cell line, the combination therapy group had a proliferation index of 63.29±1.33% compared to 80.51±1.08%, 76.56±1.59%, and 86.47±1.02% for the curcumin group, radiation group and control groups, respectively (p<0.0001). In the Rh41 cell line, the combination therapy group had a proliferation index of 66.8±0.98% compared to 81.44±1.7%, 80.77±1.6% and 86.61±0.84% for the curcumin group, radiation group and control group, respectively (p<0.0001) (Fig. S5A).

The article "Curcumin Potentiates Rhabdomyosarcoma Radiosensitivity by Suppressing NF-κB Activity" was retracted in 2019. Reasons: fabricated or falsified data; manipulated images; duplicated images.

Next, we examined tumor cell apoptosis by TUNEL staining. In both cell lines, the greatest increase in apoptotic cells was found with combination therapy. In the Rh30 cell line the combination group had 18.46±1.8 apoptotic cells/1000 cells compared to 12.15±1.1, 12.14±1.4 and 8.98±1.1 apoptotic cells/1000 cells for the curcumin group, radiation group and the control groups, respectively (p<0.0001). In the RH41 cell line the combination group had 17.11±1.1 apoptotic cells/1000 cells compared to 11.67±1.09, 10.90±.85 and 9.52±0.5 apoptotic cells/1000 cells for the curcumin group, radiation group and the control group (p<0.0004) (Fig. S5B).

### Curcumin enhances the effect of radiation on tumor cell angiogenesis

We next examined tumor microvessel density by assessing CD34 immunohistochemistry. The combination therapy resulted in the greatest decrease in tumor microvessel density in both rhabdomyosarcoma xenografts. In the Rh30 cell line, combination therapy group had 20,022±2,225 CD34 pixels/hpf compared to 33,363±2,055, 37,481±2,514 and 41,245±3,225 CD34 pixels/hpf for the curcumin group, radiation group and the control group, respectively (p<0.0001) In the Rh41 cell line, the combination therapy group had 14,353±1,740 CD34 pixels/hpf compared to 34,827±2,357, 38,994±2,955 and 46,121±4,393 CD34 pixels/hpf for the curcumin group, radiation group and the control group, respectively (p<0.0007) (Fig. S5C).

### IκBα super repression sensitizes rhabdomyosarcoma tumors to radiation

Next, we established orthotopic Rh30 EV, SR-p100 and SR-IκBα xenografts. Approximately 1 month after injection, mice bearing tumors of each cell line were size-matched into 2 groups, one group was subjected to IR (n = 10) while the other served as control. Five mice in each group were sacrificed 4 hr after exposure to 10 Gy radiation to confirm suppression of NF-κΒ activity. In the control tumors and tumors derived from the p100 super-repressor expressing cells exposed to IR, there was an increase in the NF-κΒ activity, specifically in complexes containing the p50 and p65 subunits. There was no increase in the NF-κΒ activity upon radiation exposure in tumors derived from SR-IκBα expressing cells (Fig. 6A), confirming that expression of the IκBα super-repressor inhibits radiation-induced NF-κΒ activation.

The article "Curcumin Potentiates Rhabdomyosarcoma Radiosensitivity by Suppressing NF-κB Activity" was retracted in 2019. Reasons: fabricated or falsified data; manipulated images; duplicated images.

**Figure 6:** Effects of radiation on xenografts stably expressing p100 and IκBα super-repressors. (A) EMSA revealed that radiation treatment induced NF-κB activity in tumors with empty vector and expressing p100 super-repressor, but there was no induction of NF-κB activity in tumors that expressed IκBα super-repressors. (B) Tumors expressing SR-IκBα were more sensitivity to radiation therapy than tumors with empty vector or SR-p100.

At the end of two weeks, the remaining animals were sacrificed. Tumors derived from IκBα-SR cells were 94% smaller when IR was given, compared untreated xenografts (mean tumor volume  = 62.4±10.8 mm^3^ vs. 1,019±61 mm^3^, p<0.0003). Tumors with empty vector treated with IR had a mean tumor volume of 967±64.6 mm^3^ that was only 27% less than the mean tumor volume of 1,331±133 mm^3^ in mice that did not receive radiation. Similarly, tumors derived from the p100-SR expressing cells when treated with IR, had a volume of 790±133mm^3^, which was only 30% less than the mean tumor volume of 1,125±109 mm^3^ in mice not receiving IR (Fig. 6B).

## Discussion

Radiation therapy is a critical component of the multimodality approach to the treatment of many solid tumors, including rhabdomyosarcoma. However, evidence suggests that activation of NF-κΒ, a nuclear factor involved in critical cell survival signaling pathways, can not only contribute to cancer development and progression but also mediates resistance to radiation therapy. Thus, inhibition of NF-κΒ activity has the potential to sensitize tumor cells to IR.

In the two alveolar rhabdomyosarcoma cell lines used in our study, IR upregulated NF-κΒ activity in both a time (maximally at 2 hours) and dose (10 Gy) dependent manner. Supershift assays performed with antibodies directed to specific NF-κΒ subunits showed that the p50 and p65 subunits comprised the radiation-induced NF-κΒ complex. We confirmed that IR-mediated induction of NF-κΒ activity occurred via the classical pathway in experiments with enforced expression of super repressor constructs which showed abrogation of radiation-mediated NF-κΒ activation in cell lines transduced with an SR-IκBα mutant (canonical) but not an SR-p100 (non-canonical) mutant.

Treatment with curcumin, a naturally occurring inhibitor of NF-κΒ activity, prior to the delivery of ionizing radiation, inhibited the upregulation of NF-κΒ activity in the ARMS cell lines and xenografts in response to IR, as demonstrated by EMSA. This in turn led to increased IR-mediated tumor cell apoptosis and antitumor efficacy. Activation of the classical NF-κΒ pathway is normally achieved by phosphorylation and subsequent degradation of IκBα, a cytoplasmic protein that binds and inactivates NF-κΒ by preventing its translocation into the nucleus. In our study of ARMS xenografts treated with curcumin prior to ionizing radiation, curcumin prevented the degradation of IκBα, by inhibiting the formation of the activated form of IκBα (phospho-IκBα).

The article "Curcumin Potentiates Rhabdomyosarcoma Radiosensitivity by Suppressing NF-κB Activity" was retracted in 2019. Reasons: fabricated or falsified data; manipulated images; duplicated images.

The timing of curcumin administration was critical to its radiosensitization effect as its ability to effect NF-κΒ inhibition prior to the administration of ionizing radiation was essential. We found maximal induction of NF-κΒ activation two hours after the delivery of ionizing radiation to ARMS cells *in vitro*. We did not perform time course experiments *in vivo* in our xenograft model but did find improved antitumor activity when mice were treated with curcumin for one week prior to the delivery of ionizing radiation as compared to when both were given concomitantly.

In addition to demonstrating that blocking activation of NF-κΒ by curcumin resulted in IR-mediated induction of NF-κΒ-responsive genes involved in cell proliferation (cyclin D1) and survival (XIAP and bcl-2), we showed that the combination of curcumin and IR caused a profound decrease in microvessel density in rhabdomyosarcoma xenografts. Thus, the mechanism of synergy between curcumin and IR is likely to be multifactorial and involves direct tumor cell cytotoxicity, inhibition of angiogenesis as well as radiosensitization.

One of the disadvantages of curcumin for use in the clinical setting is its limited solubility. We have overcome this problem by using liposomal curcumin. Our *in vivo* study with this formulation showed it to be well-tolerated and therapeutic doses should be easily achieved.

This is the first study, to our knowledge, that demonstrates the adjuvant antitumor activity of curcumin in vivo against rhabdomyosarcoma tumors treated with radiation therapy. In addition, we have shown that this in vivo radiosensitization is due to the abrogation of the increase in the NF-κB activity that occurs in these solid tumors in response to ionizing radiation via the classical pathway. We further confirmed these findings through suppressing NF-κB activation by genetic means. These data suggest that preventing the radiation-induced activation of the NF-κΒ pathway is a promising way to improve the antitumor efficacy of adjuvant ionizing radiation and warrants study in clinical trials.

The article "Curcumin Potentiates Rhabdomyosarcoma Radiosensitivity by Suppressing NF-κB Activity" was retracted in 2019. Reasons: fabricated or falsified data; manipulated images; duplicated images.

## Supporting Information

Figure S1 **Effects of curcumin, radiation and combination therapy on rhabdomyosarcoma tumor cell proliferation.** (A) Curcumin treatment resulted in a dose-dependent decrease in proliferation in both Rh30 and Rh41 cell lines. IC_50_ concentrations determined at 96 hr after treatment varied from 17.5 µM±1.92 for Rh30 and 19.3 µM±1.89 for Rh41 (B) Radiation therapy resulted in a dose-dependent decrease in proliferation in both the Rh30 and Rh41 cell lines. IC_50_ doses determined at 72 hr after treatment varied from 18.3±1.3Gy for Rh30 to 18.9±1.2Gy for Rh41. (C) The effects of combination therapy was synergistic in both cell lines. The Rh30 treatment resulted in a positive α non-additivity parameter of 5.54 with a 95% confidence interval (3.87, 7.20). The Rh41 treatment resulted in an α of 5.86 with a 95% confidence interval (4.55, 7.17).
(TIF)

Figure S2 **Effects of curcumin, radiation and combination therapy on rhabdomyosarcoma apoptosis.** Cells were treated with 10 µM liposomal curcumin (24 hr) prior to radiation exposure (10 Gy) and then analyzed for apoptosis by Annexin V staining. The combination therapy of curcumin and irradiation significantly increased apoptosis compared to control in both the Rh30 and Rh41 cell lines (p = .00003 and p = .0001, respectively).
(TIF)

Figure S3 **Curcumin inhibits radiation-induced upregulation of NF-κΒ dependent genes.** Western blot analysis revealed that radiation induced NF-κΒ dependent genes (MMP-9, XIAP, Bcl-2, Cox-2, Cyclin D1), which was suppressed by curcumin pretreatment in Rh30 and Rh41.
(TIF)

Figure S4 **IκBα super-repression sensitizes rhabdomyosarcoma to radiation in vitro.** (A) Rhabdomyosarcoma cell lines expressing the IκBα super-repressor were more sensitive to radiation compared to the cell lines expressing empty vector or p100 super-repressor. (B) The Rh30 and Rh41 SR-IκBα cell lines showed a significant increase in Annexin V positive cells compared to the cell lines expressing empty vector and SR-p100.
(TIF)

Figure S5 **Curcumin enhances the effect of radiation on tumor cell proliferation, apoptosis and angiogenesis.** Ki67, TUNEL, CD34 immunohistochemistry staining was used to analyze Rh30 and Rh41 tumors for tumor cell proliferation, apoptosis and angiogenesis, respectively (A) Combination therapy resulted in a significant decrease in tumor cell proliferation (p<0.0001 and p<0.0001, respectively), shown is representative Ki-67 staining (400X) (B) Combination therapy resulted in a significant increase in the TUNEL positive cells compared to control (p<0.0001 and p<0.0004, respectively), shown is representative TUNEL staining (400X) (C) Combination therapy resulted in a significant decrease in tumor microvessel density compared to control tumors (p<0.0001 and p<0.0007, respectively), shown is representative CD34 staining (400X).
(TIF)
